The article "Financial Market Sentiment Prediction Technology and Application Based on Deep Learning Model" was retracted in 2023. Reasons: signs of a paper mill; suspected computer-generated content; unreliable results or conclusions; concerns about the data.

# Financial Market Sentiment Prediction Technology and Application Based on Deep Learning Model

**DOI:** 10.1155/2022/1988396

**Published:** 2022-03-04

**Authors:** Yixuan Guo

**Affiliations:** Department of Business Administration, Shanghai Lixin University of Accounting and Finance, Shanghai 201209, China

## Abstract

In the real world, there are a variety of situations that require strategy control, that is reinforcement learning, as a method for studying the decision-making and behavioral strategies of intelligence. It has received a lot of research and empirical evidence on its functions and roles and is also a method recognized by scholars. Among them, combining reinforcement learning with sentiment analysis is an important theoretical research direction, but so far there is still relatively little research work about it, and it still has the problems of poor application effect and low accuracy rate. Therefore, in this study, we use the features related to sentiment analysis and deep reinforcement learning and use various algorithms for optimization to deal with the above problems. In this study, a sentiment analysis method incorporating knowledge graphs is designed using the characteristics of the stock trading market. A deep reinforcement learning investment trading strategy algorithm for sentiment analysis combined with knowledge graphs from this study is used in the subsequent experiments. The deep reinforcement learning system combining sentiment analysis and knowledge graph implemented in this study not only analyzes the algorithm from the theoretical aspect but also simulates data from the stock exchange market for experimental comparison and analysis. The experimental results illustrate that the deep reinforcement learning algorithm combining sentiment analysis and knowledge graphs used in this study can achieve better gains than the existing traditional reinforcement learning algorithms and has better practical application value.

## 1. Introduction

Reinforcement learning is a commonly used framework as a way to handle sequential decision-making tasks. On the other hand, deep learning can be used for the representation and storage of feature aspects [1]. So far, the combination of these two different models is by far the best answer in terms of learning good state representations of very challenging tasks that are designed to solve not only simulated scenario domains but actually challenging real-world problems. Reinforcement learning, as a subset of machine learning, which in turn is an important branch of artificial intelligence, has gained more and more importance in the last years [2]. The classical approach to creating AI requires programmers to manually code every rule that defines the behavior of the software [3]. A clear example is Stockfish, an open-source AI chess engine developed with the help of hundreds of programmers and chess experts who translated their experience into the rules of the game [4]. In contrast to rule-based AI, machine learning programs develop their behavior by examining large amounts of example data and finding meaningful correlations.

The article "Financial Market Sentiment Prediction Technology and Application Based on Deep Learning Model" was retracted in 2023. Reasons: signs of a paper mill; suspected computer-generated content; unreliable results or conclusions; concerns about the data.

In creating a machine learning-based chess engine, instead of providing rules for each game, engineers created a basic algorithm and trained it using data collected from thousands of games played by human chess players [5]. The AI model would scrutinize the data and identify similarities between winners. When offered a new game, the AI will decide on the moves most likely to lead to a win based on examples it has previously seen. While machine learning and its more advanced subset deep learning can solve many problems previously thought to be infeasible for computers, they rely on large amounts of annotated, quality training data. This limits their application to areas where labeled data are scarce [6]. This is where reinforcement learning comes into play. Humans and higher animals are able to engage in continuous interaction with their external environment to understand, explore, and sense it. This is due to the fact that humans and higher animals have the ability to continuously learn, to continuously learn and accumulate experience, and to reuse existing experience to make current decisions more rational and superior. The implication of machine learning is that machines have the same learning and perceptual capabilities as humans and can mimic the action habits of humans or higher animals in continuous interaction [7]. Machine learning has a number of advantages over human learning, and it has been shown that machine-based knowledge far exceeds the capabilities of the human brain in terms of memorizing knowledge, understanding, and comprehension. As a result, humans tend to rely more and more on machine-based knowledge. The value of utilizing machine learning in finance is becoming increasingly evident. As banks and other financial institutions strive to enhance security, streamline processes, and improve financial analysis, machine learning is becoming the technology of choice [8]. While it is true that traditional finance is not at the forefront of adopting machine learning, its use in finance is now a hit. It offers new technological services for financial forecasting, customer service, and data security. Profitable stock trading strategies are vital for investment firms [9]. It is used to optimize capital allocation, thus allowing for the maximum utilization of performance, such as expected returns. Earning maximization is based on an estimate of the potential return and risk of the stock. However, it is challenging for analysts to consider all relevant factors in a complex stock market [10].

The article "Financial Market Sentiment Prediction Technology and Application Based on Deep Learning Model" was retracted in 2023. Reasons: signs of a paper mill; suspected computer-generated content; unreliable results or conclusions; concerns about the data.

In the strategy of this study, first, the covariance matrix of expected stock returns and stock prices is calculated. Then, the optimal portfolio allocation is found by maximizing the return for a fixed risk of the portfolio or minimizing the risk for a range of returns. The optimal trading strategy is then extracted by following the optimal portfolio allocation. However, implementing this method can be very complex if the manager wants to modify the decisions made at each time step and consider the transaction costs. The process of stock investment trading can be thought of as a Markov decision process (MDP). Then, we formulate the trading objective as a maximization problem. Considering the stochastic and interactive nature of the trading market, the problem formulation of stock trading, we solve the stock trading problem by considering the stock trading process as a Markov decision process (MDP) and calculate the optimal strategy through dynamic programming ideas. However, the scalability of the model is limited by the huge state space in dealing with the stock market. In this study, however, our work is a study of stock market sentiment analysis and investment strategy algorithms based on deep reinforcement learning, which first uses knowledge mapping techniques to improve the relevance of news headlines, uses them in sentiment analysis to derive the sentiment coefficients of the corresponding stocks for each news item, and applies them to a modified deep recurrent Q-learning network (DRQN) to find the optimal trading strategy in a complex and dynamic stock market.

## 2. Related Work

In recent years, various methods based on deep reinforcement learning have been used to deal with various types of decision problems. Although the scheme of using deep learning and reinforcement learning in unison has been used in the past, deep reinforcement learning actually got a start in terms of both quality and efficiency after DeepMind proposed the DQN (deep Q network) algorithm, which accomplished the result of playing Atari games using only pure images as input and using a training intelligence throughout [11]. DeepMind then published a modified version of the previously proposed DQG in nature, which was noticed by the academic community, and it is because of this opportunity that deep reinforcement learning has gradually become a cutting-edge research in the direction of deep learning. Most of these reinforcement learning methods can be further divided into model-free-based reinforcement learning and model-based reinforcement learning [12]. In model-free-based reinforcement learning algorithms, the algorithms are able to be applied in several ways. Since it is not necessary to construct a model, all decision-making studies of intelligence are obtained by interacting with the environment [13]. Among the representative methods are Q-learning and some of its improved versions, the Monte Carlo method.

The article "Financial Market Sentiment Prediction Technology and Application Based on Deep Learning Model" was retracted in 2023. Reasons: signs of a paper mill; suspected computer-generated content; unreliable results or conclusions; concerns about the data.

Without a model, the intelligence needs to explore the external environment by interacting with the system with information all the time and training the model with a lot of trial-and-error experience in the process [14]. This is actually one of the drawbacks of model-free reinforcement learning algorithms: the efficiency of using data for simulation is too low. For these reasons, model-free-based reinforcement learning algorithms usually require millions of explorations and environments. With the above analysis, model-free-based reinforcement learning methods are actually like violent exploration, but model-free-based reinforcement learning methods are guided by the strategy of violent search [15]. Moreover, model-free-based reinforcement learning methods tend to be poorly robust, and especially after the external market environment and training work tasks change and evolve, the intelligence can generally ask us to retrain and explore [16]. Model-free methods can directly learn from experience, meaning that they can perform actions in the real world (e.g., robots) or in computers (e.g., games). They then collect rewards (either positive or negative) from the environment and update their value function. This is the main difference with model-based approaches.

The model-free approach works in the real environment for learning. Instead, the model-based algorithm reduces the interaction with the real environment during the learning phase [17–19]. The goal is to build models based on these interactions with the environment and then use that model to simulate other events. Rather than in the actual environment, it is applied to construct the model and obtain the results returned by that model. As mentioned earlier, this has the advantage of accelerated learning, as there is no need to wait for the environment to respond or to reset the environment to some state to resume learning. However, the downside is that if the model is not accurate, we risk completely learning something different from reality. Learning a model involves performing operations in a real environment and collecting feedback [20, 21]. We call this experience. Thus, for each state and action, the environment provides new states and rewards. Based on these experiences, we try to derive models, which are nothing but supervised learning problems. There are also methods that learn models with the help of neural networks and optimize reinforcement learning methods based on models using traditional theories of optimal trajectories. Such algorithms include those proposed by Levine at Berkeley and Abbeel at OpenAI. Creating a probabilistic model of the system, using a Gaussian process or probabilistic neural network to learn the model, and using the probabilistic model in planning are approaches such as the PILCO family of algorithms, mainly proposed by Rasmussen et al. in the Machine Learning Laboratory at Cambridge University.

The article "Financial Market Sentiment Prediction Technology and Application Based on Deep Learning Model" was retracted in 2023. Reasons: signs of a paper mill; suspected computer-generated content; unreliable results or conclusions; concerns about the data.

In the model-based reinforcement learning methods, if we can define our own cost function, we can apply the model to compute the optimal operation. Control theory has a strong influence on model-based RL [22]. Recent advances in model-free reinforcement learning demonstrate the ability of rich value function approximators to master complex tasks [23]. Dai and Kong pointed out that the multivariate forecasting method can greatly improve the forecasting ability of bond yield [24]. However, these model-free methods require access to an impractically large number of training interactions for most real-world problems. In contrast, model-based reinforcement learning methods can use learned models to quickly achieve near-optimal control under rather restricted classes of dynamics. In environments with nonlinear dynamics, the complex dynamics in model-based reinforcement learning methods require high-volume models, which in turn tend to be overfitted [25–28]. The two forms of reinforcement learning methods have distinct advantages and disadvantages: the expression value estimation model-free methods achieve good asymptotic performance but poor sample complexity, while the modeled methods exhibit learning with good results but struggle with complex tasks.

## 3. Knowledge Graph-Based Sentiment Analysis of the Stock Market

### 3.1. System Design

The framework of the knowledge graph-based sentiment analysis system for the stock investment market implemented in this study contains three main modules, knowledge graph module, embedding layer module, and recurrent convolutional neural network (RCNN) module. Relevant news headlines are identified at the top of the website and preprocessed using natural language processing techniques such as removing HTML tags, marking sentences, removing banned words, and so on. Subsequently, the knowledge graph is built by putting the relevant information of the stock corresponding companies, and the preprocessed news headlines are put into the knowledge graph for distance comparison. The news headlines with appropriate distances are filtered in the knowledge graph as the input of the embedding layer module, and then, the sentiment results are output through the sentiment analysis module after vectorizing the text data in the embedding layer. The specific algorithm flow is structured in Figure 1 below.

The article "Financial Market Sentiment Prediction Technology and Application Based on Deep Learning Model" was retracted in 2023. Reasons: signs of a paper mill; suspected computer-generated content; unreliable results or conclusions; concerns about the data.

The technical development routes for constructing knowledge graphs can be generally divided into two types, one of which is top-down while the other is bottom-up. One of the top-down solutions for constructing a knowledge graph is to find information such as ontologies and relationships from inside the good data and append it to the knowledge base with the help of structured data sources such as encyclopedias. The bottom-up approach to build the knowledge graph is to use specific guidelines to collect data from public resource models to obtain highly reliable information to add to the base knowledge. The knowledge graph constructed in this chapter is based on the cloning of web resources as data input, and therefore, a bottom-up approach to constructing a knowledge graph is used. The input data may be structured, unstructured, or semistructured, and based on this information data we can apply mainly our own set of systematic automated or semiautomated technical research solutions to obtain the elements of relevant knowledge, i.e., the physical-economic relationships with each other, from the very first data, and then place them in the module layer above the corresponding knowledge base and in the data layer. The construction of the knowledge graph as a process of cyclic change changes by obtaining the relationships of knowledge, and each iteration contains three stages: (1) knowledge extraction: the mutual relationships that exist inside the entities, attributes, and entities are obtained in each data source, and the dynamic knowledge representation is formed based on this logic; (2) knowledge integration: in order to obtain new knowledge after eliminating contradictions and ambiguities such as some entities can be more than one expression, there exists the possibility of some special calls corresponding to a different number of entities; (3) knowledge processing: quality assessment of new knowledge can be placed after their integration before the ranking part of the knowledge base to ensure the quality of the knowledge base. There are two possible problems with the use of remote supervision in relational extraction. First, the knowledge base and the text will use heuristic alignment in remote supervision, which may lead to errors in the annotation of the data. Second, in previous methods, specific features are used in statistical models to achieve classification, but the noise caused by specific features sometimes produces bad results. In this study, multiple example learning and PCNNs are applied to deal with the above two problems.  Figure 2 shows the structure of PCNNs.

The article "Financial Market Sentiment Prediction Technology and Application Based on Deep Learning Model" was retracted in 2023. Reasons: signs of a paper mill; suspected computer-generated content; unreliable results or conclusions; concerns about the data.

### 3.2. Market Sentiment Model Construction

After determining the direction and class of the relationship, we represent the relationship as a form of three tuples (*h*, *r*, *t*). *h* and *t* represent the head and tail entities (firms), respectively, and *r* represents the relationship between the head and tail entities. For example, (Company A, AG, Company B) indicates that Company A holds Company B. After placing the triples into the Neo4j database, the construction of the knowledge graph is completed. The use of vector form to represent the knowledge graph can be developed to make it more convenient for various social workers afterward; therefore, the goal now is to encode and compress the triad (*h*, *r*, *t*) into a low-dimensional distributed vector. After completing the construction of the knowledge graph, if new news data are directly added to the knowledge graph for relevance analysis, the ordinary Euclidean distance is difficult to meet the processing of various application requirements. In recent years, trans-series models have been widely used for knowledge representation learning of knowledge graphs. Compared with traditional training methods, trans-series models have simple parameters, are easy to train, and are less prone to these problems of overfitting.

Simply put, the relationship inside the triple instance (*h*, *r*, *t*) is compared to the interpretation from entity *h* to entity *t*. The implementation keeps adjusting *h*, *r*, and *t* (vectors of *h*, *r*, *t*) so that (*h* + *r*) is as close as possible to *t*, i.e., *h* + *r* = *t*. The knowledge graph, trained with feature vectors, can better represent the relationship between knowledge from different graph databases. The news headline data used in this chapter can calculate the distance between the knowledge by inputting it into the knowledge graph for similarity comparison, which can be limited to a fixed distance as a metric for finding implicit relationships between stock companies. A distance smaller than this indicates that this news headline has a closer relationship with the corresponding stock, and there will be factors that affect the rise or fall of the stock, which can be used as input to the sentiment analysis module. News headlines that exceed this distance can be considered as having noisy data and are not used as input for the sentiment analysis module.

The article "Financial Market Sentiment Prediction Technology and Application Based on Deep Learning Model" was retracted in 2023. Reasons: signs of a paper mill; suspected computer-generated content; unreliable results or conclusions; concerns about the data.

The word vector output from the text data after the embedding layer can be used as the input to the sentiment analysis module. The sentiment analysis model network in this chapter has three layers, i.e., LSTM (recursive) layer, convolutional layer, and output layer. The first layer is the RNN implemented as (LSTM). The LSTM layer introduces the stored elements into the network. This layer is very effective in extracting sentence representations, allowing our model to analyze long sentences. The input gate directs the amount of change in the input vector of the current time LSTM unit to the messages in the memory model, the forgetting gate acts as the degree of influence of the previous moment's history on the messages in the current time memory unit, and the output gate controls the amount of output of the messages in the memory unit. The input gate, output gate, and forgetting gate are denoted as *it*, *ot*, and *ft* below.

The second layer creates a convolution kernel that convolves with the input in a single spatial dimension to generate a tensor. This layer is used for a one-dimensional maximum pool of pool length four. This layer extracts semantic information from the word embeddings provided by the embedding layer. Where said convolution window has a large interference of size etc., similar to the selection to achieve the final classification result of the selected local feature *n* words, then the representation in the contextual semantic information, i.e., full-text semantic embodiment, is obtained. A convolutional operation window is set to carry out a size of *a* ∗ *b*, the number of words within the window is a, and the word vector space dimension is *b*. Multiple convolutional kernels are applied to generate a feature map, then, a maximum pooling layer operation is implemented, and finally, softmax is run to perform the classification.

### 3.3. Deep Learning for the Decision Process

Markov decision process, or MDP for short, has been used by a large number of researchers as a general architecture used to solve most reinforcement learning problems and to initiate subsequent theoretical research. The Markov decision process is explained by means of a 5-tuple (*S*, *A*, *P*, *R*, and *γ*), where *Z* is the set of states, which is finite in number, *B* is the set of actions, which is also is finite, *P* is the state transfer probability from one current state to the next, *R* is the reward function in the network, and *γ* is the discount rate for each cumulative calculation that can be used to calculate the cumulative reward, as shown in Figure 3.

The state transfer probability of the MDP is

(1) $$\begin{array}{c} {\tilde{A}}_{x_{II}}=\sum_{i=1}^{q}\chi_{\text{ii}}\;\Leftrightarrow \;\mu_{A}\left(x\right)=0. \end{array}$$

The meaning refers to the map from the operational state of the strategy to the notation used to represent the strategy *π*, which refers to the chosen state when *Z*, in the presence of the set of assigned actions, can be expressed as follows:

(2) $$\begin{array}{c} \tilde{A}=\tilde{B}=\sum_{i=1}^{q}\mu_{\text{ii}}\left(x\right)\;\Leftrightarrow \;\mu_{A}\left(x\right)=0. \end{array}$$

This system is fully visible inside the MDP, which means that the observation is in the same state as the environment: *ωt*=*st*. At each time step *t*, the probability of moving to *zt* + 1 is given by the state transition function *T*(*zt*, *bt*, *zt* + 1), and the reward is given by the bounded reward function *R*(*zt*, *bt*, *zt* + 1) ∈ ℛ. At each step, the intelligence takes action to change its state in the environment and provide a reward.

(3) $$\begin{array}{c} W_{i+1}=W_{i}-a\frac{\partial L}{\partial q}. \end{array}$$

The specific meaning of decision-making is available by learning conditions for the probability distribution. Decision-making in reinforcement learning is generally stochastic, and the benefit of using stochastic decisions is the ability to integrate search into the sampling step. Search here is where the intelligence goes through other actions to arrive at a better decision. In practice, various kinds of noise are prevalent, which tend to obey a normal distribution curve, and how to reduce this noise also requires the use of probabilistic aspects of the theory. The goal of reinforcement learning is to find the best decision, and through this best decision found to continue the search for the corresponding best reward, where the best is the one that maximizes the total reward in the end. The cumulative reward is defined.

(4) $$\begin{array}{c} V_{\text{map}}=\frac{\left\{a_{1},a_{2},a_{3},\ldots ,a_{n}\right\}}{\max P\left(X,Y\right)}. \end{array}$$

Under different decisions and environments, the value of *G* is uncertain. Since it is simulated under a stochastic decision *π*, the cumulative reward is also stochastic. However, the reward *E* is a value that can be determined by and we are able to perform an interpretation of the state value function. Such a function can represent the state values: when said decision agent is used by *π*, the cumulative reward can be seen as an allocation, in which *E* denotes the cumulative value returned by the *Z* state is in the equation *Z* value.

(5) $$\begin{array}{c} V_{\text{np}}=\frac{\arg v_{j}\left\{a_{1},a_{2},a_{3},\ldots ,a_{n}\right\}}{\prod P\left(X,Y\right)}. \end{array}$$

The corresponding equation for the *z* − *b* value function is

(6) $$\begin{array}{c} P_{x,y}=\frac{N\sum_{i=1}^{n}X*Y}{\sqrt{\sum_{i=1}^{n}\left(X+Y\right)}}. \end{array}$$

The Bellman equation for the *z*-valued function and the *z*-*b*-valued function are given below. From the defining equation of the *z*-valued function, it can be obtained that the Bellman equation for *z* can be expressed as

(7) $$\begin{array}{c} V_{\text{map}}=\frac{\left\{a_{1},a_{2},a_{3},\ldots ,a_{n}\right\}}{\max P\left(X,Y\right)}=P\left(X,Y\;|\;v_{j}\right)p\left(v_{j}\right). \end{array}$$

The article "Financial Market Sentiment Prediction Technology and Application Based on Deep Learning Model" was retracted in 2023. Reasons: signs of a paper mill; suspected computer-generated content; unreliable results or conclusions; concerns about the data.

## 4. Experiments and Result Analysis

### 4.1. Experimental Data and Preprocessing

Reinforcement learning is really about finding the best policy by simulating the Markov decision process of the environment and then deriving the optimal reward over the best policy by simulation. To evaluate the effectiveness of the algorithms in this chapter, a large amount of historical data on thousands of stock codes, with both outdated price information and outdated news headlines related to stock codes, is accessible using an interface provided in the financial section. This provides a rich corpus of data that can be used to train agents to correlate their interpretation of headlines with actual changes in stock prices. The site's historical data can be mined and used to train the model. It can then also be examined on a daily basis to make predictions to make predictions. Next, for each news headline, we remove the deactivated words and tokenize them. Each token is then checked for the presence of an organizational node relationship with the particular company of interest in a knowledge graph within a predetermined distance. In the experiments in this chapter, the size of the distance measure chosen is important. Choosing a walking distance longer than this would result in too much noise, while any shorter walking distance would mean that few implicit relationships would be found. The value was empirically adjusted based on conducting some manual experiments. Once any marker in the title was found to be within a predetermined distance of the stock-related organization, by extension, the entire title could be considered relevant to the organization under consideration. In this experiment, 9,463 news headlines for 100 different ticker symbols and 26,017 daily quote instances within the same time frame were collected. The raw HTML data were parsed and filtered to obtain raw tuples of <date, headline> and <date, and quote > instances, which were then sorted by date and merged to provide instances that the model could learn from. As shown in Figure 4, a particular quote instance is classified as RISE or FALL if it is up or down by more than 10% of the previous day's price; otherwise, these data are treated as “None.” The prior probabilities of RISE, FALL, or NOTHING in all collected data are 0.014672, 0.008354, and 0.987639, respectively.

The article "Financial Market Sentiment Prediction Technology and Application Based on Deep Learning Model" was retracted in 2023. Reasons: signs of a paper mill; suspected computer-generated content; unreliable results or conclusions; concerns about the data.

### 4.2. Model Training Setup and Comparison

Because the model has many variable hyperparameters and it is impractical to experiment with the optimal parameters one by one in huge parameter space, the experiments in this section use a grid search approach to perform parameter optimization. To reduce the chance of tuning the parameters for training, the experiments refer to the three-time cross-validation method. For the training process, 80% of the headlines are randomly sampled from the crawled news headline dataset as the training set, 10% of the headlines are randomly sampled as the validation set in the testing process, and the remaining 10% of the headlines are set as the test set to find the best hyperparameters by comparing the three experiments. In this experiment, 9,463 news headlines for 100 different ticker symbols and 26,017 daily quote instances within the same time frame were collected. The loss function is used for cross-entropy, and the gradient descent method for the training optimization process uses SGD stochastic gradient descent method to find the best learning rate through experiments. The results of a simple control experiment show that the best prediction results are obtained when the learning rate is 0.001. Due to the limitation of space, some of the best parameter results derived from the grid search are directly given here, which are the convolutional kernel size 64, the number of convolutional kernels is 4, the number of LSTM hidden cells is 128, the dropout retention ratio is 0.6, and the knowledge graph ontology distance is 5. On this basis, the optimal parameter comparison results for the word vector dimension are made as shown in Figure 5.

The accuracy of KGRCNN is above 86% in the best combination of hyperparameters. The experiments comparing the model in this study with other methods reveal that the KGRCNN method has a great advantage over the common LR and SVM models, while the RCNN model can classify the stock market sentiment better and simply using a CNN or RNN approach does not affect the results and the RCNN. A random sample of 90% of the data was used for training, and 10% was reserved for testing. The data chosen for training and testing are randomly selected at runtime. This assumes abstraction of any temporal information that may be present in the data that may affect classification. That is, the training instances were considered independent of each other and only dated so that citations could be matched to titles. The increased amount of training data (of which 10% was reserved for testing and not used for training) was tested against the agents. The experiments were conducted in two of them, the analysis of the prediction accuracy results of the sentiment analysis module without and with the knowledge graph technique.

The article "Financial Market Sentiment Prediction Technology and Application Based on Deep Learning Model" was retracted in 2023. Reasons: signs of a paper mill; suspected computer-generated content; unreliable results or conclusions; concerns about the data.

**Experiment 1 .**

First, the first experiment was performed using the full sentiment analysis module, on which the experiments were separately performed on the effect of using or not using the knowledge graph technique on the results of the experiments and the results are shown in Figure 6 below.

**Experiment 2 .**

The second experiment uses the knowledge graph technique but removes RNN and CNN from the sentiment analysis module, respectively, to test the effect on the results of the experiment, with the following results in Figure 7. To reduce the chance of tuning the parameters for training, the experiments refer to the three-time cross-validation method.

**Experiment 3 .**

The third experiment did not use knowledge graph techniques and removed RNN and CNN from the sentiment analysis module, respectively, to test the effect on the experimental results, which are shown in Figure 8 below.

From the above figure, it can be seen that the combined knowledge graph algorithm used in this study is enough to obtain better accuracy compared to the model without using knowledge graph techniques under the same sentiment analysis module and training data share. The sentiment analysis module using LSTM + CNN also works better than the experiments using only CNN and LSTM. The reason for this is that the internal correlation between real stocks is fully taken into account using the knowledge graph, avoiding the limitation of using only stock price data to measure correlation. RCNN can draw on the advantages of both RNN and CNN. The maximum pool extraction of the convolutional layer extracts the best representation of the input. The recurrent nature of the network captures a greater degree of pre- and post-textual information when learning text data. The accuracy, recall, F1 scores, and other results of the algorithm steadily improve as the training data increases, and we demonstrate the effectiveness of the algorithm. Based on the idea that knowledge graphs can discover implicit relationships between data, an improved research method for analyzing sentiment problems incorporating relevant knowledge graphs is implemented, and the analysis of the algorithm used in the system reveals that by simply applying a recurrent neural network (RNN) classifier for sentiment analysis, it is unable to identify distinguishing phrases that appear in different orders. In contrast, the convolutional layer can fairly identify the ambiguous phrases in the text through the maximum pooling layer. Thus, the convolutional neural network (CNN) can better reflect the context of the word as compared to RNN. The system thus chooses recurrent convolutional neural network (RCNN) as the sentiment analysis module for sentiment classification. The maximum pool extraction of the convolutional layer extracts the best representation of the input. The recurrent nature of the network will capture the preceding and following textual information in a greater possible way when learning textual representations. The final experimental results show that when the amount of training data is boosted, the accuracy of the prediction results accordingly increases.

The article "Financial Market Sentiment Prediction Technology and Application Based on Deep Learning Model" was retracted in 2023. Reasons: signs of a paper mill; suspected computer-generated content; unreliable results or conclusions; concerns about the data.

Applying the combination of deep recurrent Q networks (DRQN), prioritized experience replay mechanism, sentiment analysis, and knowledge graph to stock investment strategy research, a deep reinforcement learning algorithm PERDRQN based on deep recurrent Q networks (DRQNs) and prioritized experience replay are proposed to perform stock investment strategy research methods. Simulation experiments using deep learning libraries such as TensorFlow are conducted to verify that the algorithm proposed in this chapter can effectively perform the stock investment strategy task. The algorithm uses an end-to-end training model that combines the feature refinement and combination capabilities of deep recurrent convolutional neural networks and the good strategy formulation capabilities of reinforcement learning, which can obtain information about a stock and its company by crawling data on websites and some publicly available datasets, and after processing it through the knowledge graph and using it as input to the RCNN model, the sentiment of the company's stock is output after network processing, and then, this sentiment analysis combined with the stock information is added inside a deep reinforcement learning model to output an investment strategy. The deep recurrent Q network (DRQN) algorithm combines a convolutional neural network and a recurrent neural network to train the target value function compared to previous Q learning-based reinforcement learning algorithms, optimizing the previous Q learning scheme of training through tables or using linear regression, allowing the algorithm to represent a larger space of action states.

## 5. Conclusions

The machine has certain intelligence after using deep learning and reinforcement learning. In the process of expanding the theory and practice of machine learning, the theory and results of some disciplines have been integrated, including artificial intelligence, psychology, biology, game theory, and cybernetics, and also interact with many disciplines to get some innovative research directions. Reinforcement learning theory has become one of the hot research directions in the artificial intelligence community after years of pioneering development. However, there are still many problems that need to be improved, such as the balance between exploration and exploitation, the long training period, and the “dimensional disaster.” Because the previous work is basically gathered in theoretical research, deep reinforcement learning is relatively little applied in financial investment. In this study, we apply the deep reinforcement learning algorithm PERDRQN, which combines the sentiment analysis method of knowledge graph with the deep reinforcement learning method of prioritized experience replay, based on the study of deep reinforcement learning algorithms for stock investment strategies. Then, the technique of prioritized empirical replay is analyzed and its use in combination with DRQN reduces the time required for convergence and gives better results. The algorithm showed better results in the comparison experiments, indicating that the sentiment analysis approach combined with knowledge graphs is helpful for the deep reinforcement learning strategy framework used in this study. In the future, the accuracy, recall, F1 scores, and other results of the algorithm steadily would be improved as the training data increase.

The article "Financial Market Sentiment Prediction Technology and Application Based on Deep Learning Model" was retracted in 2023. Reasons: signs of a paper mill; suspected computer-generated content; unreliable results or conclusions; concerns about the data.

## Figures and Tables

**Figure 1:** Flowchart of knowledge graph-based sentiment analysis algorithm.

**Figure 2:** Structure of PCNNs.

**Figure 3:** Calculation of cumulative reward.

**Figure 4:** Collation of financial data.

**Figure 5:** Experimental results of tuning the optimal word vector dimension under three cross-validations.

**Figure 6:** Effect of using or not using knowledge graph technology on experimental results.

**Figure 7:** Effect of removing RNN and CNN on experimental results.

**Figure 8:** Comparison of accuracy rates in sentiment analysis.

## Data Availability

The data used to support the findings of this study are available from the corresponding author upon request.
